The article "Trastuzumab induces PUMA‐dependent apoptosis and inhibits tumor growth in gastric cancer" was retracted in 2023. Reasons: duplicated images; signs of a paper mill.

# Trastuzumab induces PUMA‐dependent apoptosis and inhibits tumor growth in gastric cancer

**DOI:** 10.1002/2211-5463.12522

**Published:** 2018-11-19

**Authors:** Linghe Luo, Haiyan Liu, Qian Xi

**Affiliations:** ^1^ Department of Gastroenterology Tongde Hospital of Zhejiang Province Hangzhou China; ^2^ Department of Radiology Shanghai East Hospital Tongji University School of Medicine Shanghai China

**Keywords:** apoptosis, gastric cancer, GC, GSK3β, PUMA, trastuzumab

## Abstract

Gastric cancer (GC) is one of the most prevalent cancers worldwide. Trastuzumab has been approved for the treatment of metastatic GC, gastroesophageal junction cancer, and breast cancer. However, the mechanisms involved in trastuzumab‐induced GC cell apoptosis remain largely unknown. In this study, we investigated the underlying mechanisms of trastuzumab‐mediated suppression of GC cell growth both *in vitro* and *in vivo*. We found that trastuzumab treatment induces p53 upregulated modulator of apoptosis (PUMA) expression in GC cells, through the NF‐κB pathway following AKT inhibition and glycogen synthase kinase 3β (GSK3β) activation. We also observed that PUMA was necessary for trastuzumab‐induced apoptosis in GC cells. Moreover, PUMA deficiency suppressed apoptosis and the antitumor effect of trastuzumab in xenograft models. Finally, computerized tomography (CT) and immunohistochemistry results showed that patients with increased activation of PUMA were more sensitive to trastuzumab treatment than those with low PUMA expression. These results indicate that trastuzumab induces PUMA‐dependent apoptosis and inhibits tumor growth in GC, suggesting that PUMA plays a critical role in mediating the antitumor effects of trastuzumab in GC. PUMA induction may be used as a marker of trastuzumab sensitivity.

**Abbreviations**
ATCC: American Type Culture Collection
CT: computerized tomography
DSCT: dual‐source computed tomography
GC: gastric cancer
GSK3β: glycogen synthase kinase 3β
HER2: human epidermal growth factor receptor 2
PUMA: p53 upregulated modulator of apoptosis
RT‐PCR: reverse transcriptase‐real‐time PCR
TFs: transcriptional factors

Gastric cancer (GC) is currently one of the most prevalent cancers worldwide 1. Unfortunately, most GC patients are diagnosed at the terminal stage of the disease 1, 2. Many patients develop metastasis even if radical excision is performed 1, 3. Remarkable progress has been made in the surgical treatment for GC, yet the 5‐year overall survival rate is limited to 24.5% in Europe and merely 40–60% in Asia. This latter finding may be attributable to an elevated recurrence rate 2. Previous studies have proved that the median survival of patients with terminal GC lacking chemotherapy is no longer than six months 4, 5. Thus far, the understanding of how chemotherapy drugs counteract malignancies is insufficient.

The article "Trastuzumab induces PUMA‐dependent apoptosis and inhibits tumor growth in gastric cancer" was retracted in 2023. Reasons: duplicated images; signs of a paper mill.

As a humanized antibody acting against human epidermal growth factor receptor 2 (HER2), trastuzumab has been approved by the FDA to treat metastatic GC, gastroesophageal junction cancer, as well as breast cancer expressing HER2 at very high levels 6, 7, 8. Although trastuzumab is effective, more than 70% of patients do not respond to the drug (de novo resistance); meanwhile, the majority of patients who do respond to trastuzumab therapies show various levels and kinds of resistance in the first year subsequent to trastuzumab treatment (acquired resistance) 9, 10. Pertuzumab is another type of humanized antibody acting against HER2. The supplementation of pertuzumab with trastuzumab remarkably postponed trastuzumab response and promoted its ability to counteract the development of subsequent malignancy 11, 12. Nevertheless, the objective response rate to this therapy is merely 24.2%, while a complete response is limited to 8% 12, 13. P53 upregulated modulator of apoptosis (PUMA), which is transcriptionally targeted by p73 and p53, can stimulate cell apoptosis in diverse malignancies 14. PUMA, which is a member of the Bcl‐2 family, possesses one ‘BH3‐only’ domain. 15. It is located in the mitochondria where it stimulates cell apoptosis when modulated by mitochondrial malfunction 16. It acts against the activities of Mcl‐1 as well as Bcl‐X_L_ via Bax/Bak 17. It has been indicated by various studies that cancer growth can be suppressed by PUMA 18. Additionally, PUMA independent of or accompanied by chemotherapy or radiotherapeutic agents displays a remarkable capacity to counteract the development of various types of malignancies 19, 20. Although trastuzumab triggers diverse reactions in HER2‐positive GC patients, the mechanisms underlying its GC inhibitory effect remain unclear.

In this study, we aimed to elucidate the mechanisms of trastuzumab involved in suppressing GC cell growth both *in vitro* and *in vivo*.

## Materials and methods

### Cell culture

Human GC line NCI‐N87 was acquired from American Type Culture Collection (ATCC, Manassas, VA, USA). DMEM was supplemented with 100 μg·mL^−1^ streptomycin, 100 units·mL^−1^ penicillin, and 10% v/v of heat‐inactivated newly born calf serum (Invitrogen, Carlsbad, CA, USA). Drugs applied to counteract malignancy such as BAY 11‐7082 (Merck, Kenilworth, NJ, USA) as well as trastuzumab (Genentech, South San Francisco, CA, USA) were dissolved in DMSO. AKT, which was constitutively activated, was obtained from Addgene (Cambridge, MA, USA).

The article "Trastuzumab induces PUMA‐dependent apoptosis and inhibits tumor growth in gastric cancer" was retracted in 2023. Reasons: duplicated images; signs of a paper mill.

### MTS

Cells (1×10^4^ cells/well) were cultured in 96‐well microtiter plates. Subsequent to overnight incubation, the wells were supplemented with the indicated dilution range of trastuzumab. Subsequently, plates were incubated for a further 72 h. Following this, cellular proliferation was determined using the MTS assay kit (Promega, Madison, WI, USA). Wallac Victor 1420 Multilabel Counter, provided by PerkinElmer, was used to detect luminescence. All measurements were made in triplicate, and assays were repeated three times.

### Reverse transcriptase‐real‐time PCR

TRIzol RNA Kit (Invitrogen) was used to purify total RNA in accordance with the manufacturer's guidelines. In order to obtain cDNA, we utilized 1 μg total RNA as template in a reaction catalyzed by SuperScript II reverse transcriptase (provided by Invitrogen and used as recommended by the manufacturer). PCRs to detect differences in expression between the indicated genes were carried out in triplicate (final volume 20 μL) using SsoFasr™ Probes Supermix (Bio‐Rad Laboratories, Hercules, CA, USA). Detection was carried out using the CFX96™ Real‐time PCR System (Bio‐Rad Laboratories) using standard thermal cycling conditions over thirty‐five amplification cycles. The relative expression of related genes was assessed using standard TaqMan Gene Expression Real‐Time PCR assays. The results were measured as threshold cycles (Ct). Comparative Ct approaches (ΔΔCt) were applied to measure the expression of the targeted transcripts, and differential expression was evaluated using 2^−ΔΔCt^ approaches.

### Western blotting

Western blotting was carried out as outlined previously 21. Antibodies applied included anti‐AKT, GSK3β, FoxO3a, and p65 with or without phosphorylation, caspase 3 and 9 subsequent to cleavage, PUMA (Abcam, Cambridge, MA, USA), cytochrome *c*, E2F1, β‐actin, Bid, Bak, Bim, lamin A/C (Santa Cruz Biotechnology, Santa Cruz), STAT1, p‐STAT1, Cox IV (Cell Signaling Technology, Beverly, MA, USA), Mcl‐1, and Bcl‐X_L_ (BD, San Jose, CA, USA).

### Apoptosis assay

Cell apoptosis was assessed using nuclear staining approaches (Hoechst 33258, Invitrogen) 22. PI (Annexin V/propidium iodide) staining was performed using both Annexin‐Alexa 488 (Invitrogen) and PI. To evaluate the release of cytochrome *C,* cytosolic fractions were separated with the help of differential centrifugation, and indicated fractions were subsequently probed by western blotting.

### Transfecting and siRNA/shRNA knockdown

Lipofectamine 2000 (Invitrogen) was used to stably transfect cells. Knockdown assays were carried out using siRNA (200 pm) prior to trastuzumab treatment. SiRNA for scrambled control, for *p65* (sc‐29410), as well as for *GSK3*β (sc‐35527) were obtained from Santa Cruz Biotechnology. Plasmid DNA permitting the expression of shRNA and including the nucleotide sequence targeted by PUMA (CCT GGA GGG TCA TGT ACA ATC TCTT) or the same plasmid vector including scrambled sequence as a negative control was used to stably transfect NCI‐N87 cells. Subsequently, 96‐well plates were seeded with cells, with the growth media supplemented with 5 μg·mL^−1^ puromycin. Western blotting was used to evaluate clones that were resistant to puromycin.

The article "Trastuzumab induces PUMA‐dependent apoptosis and inhibits tumor growth in gastric cancer" was retracted in 2023. Reasons: duplicated images; signs of a paper mill.

### Chromatin immunoprecipitation

A Chromatin Immunoprecipitation Assay Kit provided by Millipore was used for the Chromatin immunoprecipitation (ChIP) assay using anti‐p65 antibody (Cell Signaling Technology). PCR was applied to evaluate the sediment using primers (5′‐CCC GCG TGA CGC TAC GGC CC‐3′ and 5′‐GTC GGT CTG TGT ACG CAT CG‐3′) for the detection and amplification of the PUMA promoter, including the potential κB site.

### Animal models of malignancies

Experimental procedures using animals were carried out according to the ethical principles of Tongde Hospital in Zhejiang Province. Nude mice were purchased from the Experimental Animal Center of Chinese Academy of Sciences in Shanghai. *PUMA*‐KD cells and parental cells were obtained. Media (0.1 mL) containing 4 × 10^6^ cells were subcutaneously injected into the back of female nude mice whose thymus had been excised. Tumors began to grow after 7 days. Mice received a supplement of trastuzumab (daily, 3 mg·kg^−1^, twice a week). Calipers were applied to measure the volume of the tumors based on the formula of &frac12; × length × width^2^. The tumors were excised as soon as the volume reached 1.0 cm^3^. The specimens were cut and fixed with formalin (10%) before they were embedded in paraffin. Cancer slices (5‐µm ‐thick) subsequent to paraffin embedding underwent TUNEL immunostaining. Secondary antibodies conjugated to AlexaFluor‐488 (Invitrogen) were used for signal examination.

### Immunohistochemistry examination

Cancer slices were placed on slides in order to carry out immunohistochemical evaluation. Deparaffinized tumor slices were incubated in citrate buffer (pH 6.0) for 40 min at 95°C in order to recover antigens. Anti‐PUMA antibodies resuspended at a dilution of 1:100 were consequently added to these slices and incubated at room temperature for 2 h. The avidin–biotin–peroxidase complex approach was utilized to terminate immunoreactive staining.

### Computerized tomography and tissue specimens

Each computerized tomography (CT) scan was acquired using a dual‐source computed tomography (DSCT) scanner. Twenty GC patients who received trastuzumab treatment were recruited from Tongde Hospital of Zhejiang Province, China. CT was conducted prior and subsequent to treatment, in order to measure the size of the tumors. Informed consent was acquired from patients, and the Ethics Committee of Tongde Hospital of Zhejiang Province approved our study. GC specimens were obtained from patients during the course of their surgeries. Personal information of patients was maintained confidential. Every sample was pathologically analyzed and categorized in agreement with WHO criteria. The experiments were undertaken with the understanding and written consent of each subject. The study methodologies conformed to the standards set by the Declaration of Helsinki.

The article "Trastuzumab induces PUMA‐dependent apoptosis and inhibits tumor growth in gastric cancer" was retracted in 2023. Reasons: duplicated images; signs of a paper mill.

### Statistical analysis

graphpad prism iv (La Jolla, CA, USA) software was applied to conduct statistical analysis. Student's *t*‐test was used to analyze data. *P* < 0.05 indicated statistical significance. Results are presented as means ± SD.

## Results

### Trastuzumab triggered PUMA stimulation independent of p53 in GC cells

In order to explore how cell apoptosis was triggered by trastuzumab in GC cells, expression of PUMA was examined in NCI‐N87 cells supplemented with trastuzumab. Addition of trastuzumab to NCI‐N87 cells remarkably promoted transcription as well as translation of PUMA depending on dose and time (Fig. 1A–C). Transcription and translation of PUMA were also triggered by trastuzumab in *p53*‐KD NCI‐N87 cells (Fig. 1D). Trastuzumab supplement did not promote the protein level of Bim, but reduced the protein level of antiapoptotic, such as Mcl‐1 and Bcl‐X_L_ (Fig. 1E). These results indicate that trastuzumab can trigger the expression of PUMA based on p53 and that the malignancy counteraction effect of trastuzumab could be attributable to PUMA.

**Figure 1:** Trastuzumab induces p53‐independent PUMA induction in gastric cancer cells. (A) NCI‐N87 cells were treated with 10 μmol·L^−1^ trastuzumab at indicated time point. *PUMA* mRNA induction by trastuzumab was analyzed by reverse transcriptase‐real‐time (RT‐PCR), with β*‐actin* as a control. The results were expressed as the means ± SD of three independent experiments. ***P<0.001; **P<0.01 (Student's *t*‐test). (B) NCI‐N87 cells were treated with 10 μmol·L^−1^ trastuzumab at indicated time point. PUMA expression was analyzed by western blotting. (C) NCI‐N87 cells were treated with trastuzumab at indicated concentration for 24 h. PUMA expression was analyzed by western blotting. (D) NCI‐N87 cells transfected with p53 siRNA or control siRNA were treated with trastuzumab at indicated concentration for 24 h. PUMA expression was analyzed by western blotting. (E) NCI‐N87 cells treated with 10 μmol·L^−1^ trastuzumab at indicated time point. The expression of indicated Bcl‐2 family members was analyzed by western blotting.

The article "Trastuzumab induces PUMA‐dependent apoptosis and inhibits tumor growth in gastric cancer" was retracted in 2023. Reasons: duplicated images; signs of a paper mill.

### PUMA participated in cell apoptosis triggered by trastuzumab

Subsequently, the role of PUMA in cell apoptosis triggered by trastuzumab was explored using *PUMA*‐KD NCI‐N87 cells. When supplemented with trastuzumab, cell apoptosis was noticeably stimulated in NCI‐N87 cells, whereas it was considerably suppressed in *PUMA*‐KD cells (Fig. 2A). The limited expression of PUMA in NCI‐N87 cells suppressed cell apoptosis triggered by trastuzumab, which was verified using Annexin V/PI staining (Fig. 2B). Trastuzumab supplementation triggered the stimulation of caspase‐9 as well as caspase‐3, and the release of cytochrome c, which were inhibited in *PUMA*‐KD cells (Fig. 2C,D). These results show that PUMA is essential for cell apoptosis triggered by trastuzumab in GC cells.

**Figure 2:** The PUMA mediates the anticancer effects of trastuzumab through the mitochondrial pathway. (A) Parental and *PUMA*‐KD NCI‐N87 cells were treated with trastuzumab at indicated concentration for 24 h. PUMA knockdown was detected by western blotting (Left). Apoptosis was analyzed by a nuclear fragmentation assay (Right). (B) Parental and *PUMA*‐KD NCI‐N87 cells were treated with 10 μmol·L^−1^ trastuzumab for 24 h. Apoptosis was analyzed by Annexin V/PI staining followed by flow cytometry. (C) Parental and *PUMA*‐KD NCI‐N87 cells were treated with 10 μmol·L^−1^ trastuzumab for 24 h. Cleaved caspase 3 and active caspase 9 expression were analyzed by western blotting. (D) The cytoplasm and mitochondria were fractionated from parental and *PUMA*‐KD NCI‐N87 cells treated with 10 μmol·L^−1^ trastuzumab for 24 h. The distribution of cytochrome *C* was analyzed by western blotting. β*‐Actin* and cytochrome oxidase subunit IV (Cox IV) were analyzed as the control for loading and fractionation. Results in (A) and (B) were expressed as means ±SD of 3 independent experiments. **P < 0.01; *P < 0.05 (Student's *t*‐test).

### NF‐κB modulated expression of PUMA triggered by trastuzumab

The mechanisms by which PUMA was stimulated by trastuzumab were then explored. Some transcriptional factors (TFs) that modulate the stimulation of PUMA in *p53*‐KD NCI‐N87 cells were evaluated in order to reveal the mechanisms of how PUMA was stimulated. Previous works reported that Her2 inactivation promotes PUMA upregulation in FoxO3a‐dependent increase of PUMA expression, which in turn triggers apoptosis 23, 24. Our results showed that FoxO3a was not included as a result of its unaltered suppression of phosphorylation following trastuzumab supplement (Fig. 3A). STAT1 and p73 were eliminated because of a lack of stimulation in phosphorylation/activation assays (Fig. 3A).

The article "Trastuzumab induces PUMA‐dependent apoptosis and inhibits tumor growth in gastric cancer" was retracted in 2023. Reasons: duplicated images; signs of a paper mill.

**Figure 3:** p65 mediates trastuzumab‐induced *PUMA* induction. (A) NCI‐N87 cells were treated with 10 μmol·L^−1^ trastuzumab at indicated time point. Indicated protein expression was analyzed by western blotting. (B) NCI‐N87 cells were treated with 10 μmol·L^−1^ trastuzumab at indicated time point. p‐p65 (S536) and p65 expression was analyzed by western blotting. (C) NCI‐N87 cells were transfected with either a control scrambled siRNA or a *p65* siRNA for 24 h and then treated with 10 μmol·L^−1^ trastuzumab for 24 h. p65 and PUMA expression was analyzed by western blotting. (D) NCI‐N87 cells were pretreated with 10 μmol·L^−1^ BAY11‐7082 for 1 h and then with 10 μmol·L^−1^ trastuzumab for 24 h. Nuclear fractions were isolated from cells and analyzed for p65 expression by western blotting. Lamin A/C and β‐actin were used as controls for loading and fractionation. (E) NCI‐N87 cells were pretreated with 10 μmol·L^−1^ BAY11‐7082 for 1 h and then with 10 μmol·L^−1^ trastuzumab for 24 h. p‐p65 (S536) and PUMA expression was analyzed by western blotting. (F) Chromatin immunoprecipitation (ChIP) was performed using anti‐p65 antibody on NCI‐N87 cells following trastuzumab treatment for 12 h. ChIP with the control IgG was used as a control. PCR was carried out using primers surrounding the p65 binding sites in the *PUMA* promoter.

It was previously reported that NF‐κB participated in PUMA transcription after the addition of Aurora kinase inhibitors 17, TNF‐α, or regorafenib 25. NCI‐N87 cells receiving trastuzumab triggered *p65* (S536) phosphorylation in a time‐dependent manner (Fig. 3B). PUMA stimulation was inhibited by *p65* knockdown with the help of siRNA via supplementation with trastuzumab (Fig. 3C). Subsequently, *p65* was translocated to the nucleus, which could be inhibited by the specific suppressor of NF‐κB, BAY 11‐7082 (Fig. 3D). NF‐κB suppression eliminated stimulation of PUMA as well as phosphorylation of p65 triggered by trastuzumab, indicating that p65 stimulation/nuclear translocation modulated PUMA promotion via trastuzumab (Fig. 3E). Consequently, the ability of NF‐κB to bind to the promoter of PUMA was explored. It was discovered by ChIP that *p65* was recruited to the PUMA promoter after the addition of trastuzumab (Fig. 3F). Thus, our research proved that the expression of PUMA was modulated by p65 via direct binding to various κB sites as a result of trastuzumab supplementation.

### GSK3β is necessary for PUMA activation by trastuzumab

Subsequently, we determined whether GSK3β participated in the stimulation of p65 triggered by trastuzumab. First, we found that *GSK3*β siRNA but not the control siRNA suppressed trastuzumab‐induced nuclear translocation of p65 (Fig. 4A). GSK3β exhaustion eliminated PUMA stimulation triggered by trastuzumab in NCI‐N87 cells (Fig. 4B). Supplementation with trastuzumab remarkably inhibited AKT (Ser473) stimulation in a time‐dependent manner (Fig. 4C). Furthermore, treatment with trastuzumab inhibited GSK3 β Ser9 phosphorylation, which inhibited its kinase activity (Fig. 4C). Excessive expression of AKT that was constitutively activated in turn inhibited stimulation of PUMA as well as p65 triggered by trastuzumab (Fig. 4D). Our research indicates that AKT suppression modulated stimulation of GSK3β, bringing about translocation of p65 as well as stimulation of PUMA via trastuzumab.

The article "Trastuzumab induces PUMA‐dependent apoptosis and inhibits tumor growth in gastric cancer" was retracted in 2023. Reasons: duplicated images; signs of a paper mill.

**Figure 4:** The PUMA induction by trastuzumab is mediated through GSK3β activation. (A) NCI‐N87 cells were transfected with either a control scrambled siRNA or a *GSK3*β siRNA for 24 h and then treated with 10 μmol·L^−1^ trastuzumab for 6 h. Nuclear fractions were isolated from cells treated with trastuzumab and analyzed for p65 and GSK3β expression by western blotting. (B) NCI‐N87 cells were transfected with either a control scrambled siRNA or a *GSK3*β siRNA for 24 h and then treated with 10 μmol·L^−1^ trastuzumab for 24 h. GSK3β and PUMA expression was analyzed by western blotting. (C) NCI‐N87 cells were treated with 10 μmol·L^−1^ trastuzumab at indicated time point. Relative protein expression was analyzed by western blotting. (D) NCI‐N87 cells were transfected with active AKT plasmid for 8 h and then treated with 10 μmol·L^−1^ trastuzumab for 24 h. PUMA, p‐AKT, and total AKT expression was analyzed by western blotting.

### PUMA participated in malignancy counteraction of trastuzumab *in vivo*

Whether cell apoptosis was modulated by PUMA participating in trastuzumab‐mediated counteraction of malignancy was then explored in xenografts, which were generated with the help of *PUMA*‐KD as well as parental NCI‐N87 cells in nude mice. Mice developing cancer received trastuzumab (3 mg·kg^−1^) or vehicle twice a week. The size of the tumors was examined every 48 h. *PUMA*‐KD, as well as parental tumors, displayed nearly identical growth patterns in groups without trastuzumab supplementation. Parental cancer growth was inhibited by 70–80% trastuzumab supplement (Fig. 5A). Contrarily, *PUMA*‐KD tumors displayed weaker growth suppression subsequent to trastuzumab supplementation in comparison with parental cancers (Fig. 5A), suggesting that PUMA shortage eliminated trastuzumab‐mediated counteraction of malignancy. Trastuzumab promoted the expression of PUMA as well as phosphorylation of p65 in xenografts (Fig. 5B). It was suggested by TUNEL staining that cell apoptosis was noticeably promoted in parental cancers when supplemented with trastuzumab. However, TUNEL staining of *PUMA*‐KD cancers supplemented with trastuzumab (Fig. 5C) was not positive. Consequently, our results indicate that PUMA was essential for trastuzumab‐mediated counteraction of malignancy *in vivo*.

The article "Trastuzumab induces PUMA‐dependent apoptosis and inhibits tumor growth in gastric cancer" was retracted in 2023. Reasons: duplicated images; signs of a paper mill.

**Figure 5:** The PUMA mediates the antitumor effects of trastuzumab in a xenograft model. (A) Nude mice were injected s.c. with 4 × 10^6^ parental and *PUMA*‐KD NCI‐N87 cells. After 1 week, mice were treated with 3 mg·kg^−1^ trastuzumab or buffer. Tumor volume at indicated time points after treatment was calculated and plotted (*n* = 7 in each group). Results were expressed as means ± SD of 3 independent experiments. **P < 0.01; *, *P* < 0.05 (Student's *t*‐test). (B) Parental NCI‐N87 xenograft tumors were treated with 3 mg·kg^−1^ trastuzumab or the control buffer as in (A). Phospho‐p65 (S536) and PUMA in representative tumors were analyzed by western blotting. (C) Paraffin‐embedded sections of tumor tissues from mice treated as in (A) were analyzed by TUNEL staining. Representative staining pictures (left) and TUNEL‐positive cells (right) were counted and plotted. Scale bar, 50 μm. Results were expressed as means ± SD of 3 independent experiments. **P < 0.01 (Student's *t*‐test).

### PUMA determines trastuzumab sensitivity in GC patients

In order to assess the role of PUMA in trastuzumab sensitivity in GC patients, twenty GC patients who had received trastuzumab therapy were studied. The size of each tumor was examined by using CT prior and subsequent to trastuzumab supplement. Immunohistochemical and RT‐PCR analyses were used to detect PUMA expression. Additionally, PUMA expression and alterations in cancer sizes in twenty GC tissues were examined using RT‐PCR and CT. Our study showed that the expression of PUMA was linked with cancer size suppression (Fig. 6A,B), indicating that the expression of PUMA served as a reliable predictor of trastuzumab sensitivity in treatment of GC.

**Figure 6:** The PUMA as a biomarker of trastuzumab sensitivity in gastric cancer patients. (A) Gastric biopsy samples were obtained from patients. Immunohistochemistry was performed on specimens using anti‐PUMA. Scale bar, 100 μm. (B) PUMA expression was found to be associated with tumor volume change by analyzing 20 independent gastric tissues.

## Discussion

Developing drug resistance remains the first challenge of antitumor treatment 26, 27. Furthermore, when the occurrence of breakdowns in the normal functioning of shared molecular pathways triggers carcinogenesis, the choice of antitumor treatments can be greatly complicated 28, 29. Our research aimed at revealing the link between expression of PUMA and trastuzumab‐mediated mechanisms of counteracting malignancy in GC. In our study, the role of trastuzumab in GC was explored. Our findings are the first to demonstrate that trastuzumab‐mediated mechanisms of counteracting malignancy are modulated by autonomic cell apoptosis, which results from AKT suppression, nuclear translocation of p65, as well as GSK3β stimulation, thereby bringing about PUMA stimulation and mitochondrial‐dependent cell apoptosis. Our results indicate that trastuzumab induces PUMA‐dependent apoptosis and inhibits tumor growth in GC, suggesting that PUMA plays a critical role in mediating the antitumor effects of trastuzumab in GC and PUMA induction may be used as an indicator of trastuzumab sensitivity.

The article "Trastuzumab induces PUMA‐dependent apoptosis and inhibits tumor growth in gastric cancer" was retracted in 2023. Reasons: duplicated images; signs of a paper mill.

Illuminating the response to trastuzumab remains an essential challenge in order to treat GC patients not responding to trastuzumab‐dependent chemotherapy, because HER2 serves as a promising target of GC cells that are HER2 positive. Until now, the roles played by individual contributors to the trastuzumab response are not sufficiently well understood. However, it has been discovered that trastuzumab sensitivity is linked to excessive expression of HER2 in diverse malignancies. Previous study demonstrated that HER2 directly phosphorylates PUMA and this leads to PUMA degradation and suppression of apoptosis 30. In our research, we demonstrated that the expression of PUMA is triggered by trastuzumab via the GSK‐3β/NF‐κB pathway subsequent to AKT suppression and triggers cell apoptosis depending on the number of mitochondria in GC cells. PUMA stimulation is involved in cell apoptosis brought about by chemotherapeutic drugs and serves as a promising predictor of sensitivity. It has been demonstrated in a previous study that PUMA stimulation is linked with diverse EGFR TKIs sensitivity and that insufficient PUMA stimulation is linked with EGFR TKI resistance 31. Additionally, it has been recently reported that the reaction of separated mitochondria from mutations to BH3 domains of PUMA is related to chemotherapy response 31, 32, 33. The findings of our study indicate that the expression of PUMA can serve as a reliable predictor of malignancy counteraction of trastuzumab in GC cells. Despite the fact that acquiring biopsies from GC patients receiving chemotherapy following surgery is difficult, it is nonetheless a promising line of inquiry to examine PUMA stimulation in noninvasive ways, including evaluation of cancer cells in circulation.

## Conclusions

In conclusion, our study elucidated an innovative way in which malignancy can be counteracted using trastuzumab, via cell apoptosis modulated by PUMA, independent of p53. Furthermore, trastuzumab‐mediated alterations in PUMA expression may serve as a reliable predictor in clinical experiments and can assist in determining essential implications for therapeutic progression as well as for applications in the future.

The article "Trastuzumab induces PUMA‐dependent apoptosis and inhibits tumor growth in gastric cancer" was retracted in 2023. Reasons: duplicated images; signs of a paper mill.

## Author contributions

HL and QX conceived and designed the project. LL, HL, and QX performed the experiments. LL and QX wrote the manuscript. HL and QX revised the final manuscript.

## Conflict of interest

The authors declare no conflict of interest.

## References

[1] Hu B , El Hajj N , Sittler S , Lammert N , Barnes R and Meloni‐Ehrig A (2012) Gastric cancer: classification, histology and application of molecular pathology. J Gastrointest Oncol 3, 251–261.2294301610.3978/j.issn.2078-6891.2012.021PMC3418539

[2] Carcas LP (2014) Gastric cancer review. J Carcinog 13, 14.2558989710.4103/1477-3163.146506PMC4278094

[3] Ajani JA , Lee J , Sano T , Janjigian YY , Fan D and Song S (2017) Gastric adenocarcinoma. Nat Rev Dis Primers 3, 17036.2856927210.1038/nrdp.2017.36

[4] Li S , Lan X , Gao H , Wang W , Chen L , Song S and Xue Y (2017) Addition of peritonectomy to gastrectomy can predict good prognosis of gastric adenocarcinoma patients with intraoperatively proven single P1/P2 carcinomatosis. Tumour Biol 39, 1010428317697567.2861895710.1177/1010428317697567

[5] Zali H , Rezaei‐Tavirani M and Azodi M (2011) Gastric cancer: prevention, risk factors and treatment. Gastroenterol Hepatol Bed Bench 4, 175–185.24834180PMC4017429

[6] Garnock‐Jones KP , Keating GM and Scott LJ (2010) Trastuzumab: A review of its use as adjuvant treatment in human epidermal growth factor receptor 2 (HER2)‐positive early breast cancer. Drugs 70, 215–239.2010899310.2165/11203700-000000000-00000

[7] Sakai D , Satoh T , Kurokawa Y , Kudo T , Nishikawa K , Oka Y , Tsujinaka T , Shimokawa T , Doki Y and Furukawa H (2013) A phase II trial of trastuzumab combined with irinotecan in patients with advanced HER2‐positive chemo‐refractory gastric cancer: Osaka Gastrointestinal Cancer Chemotherapy Study Group OGSG1203 (HERBIS‐5). Jpn J Clin Oncol 43, 838–840.2385264810.1093/jjco/hyt083

[8] Sanford M (2013) Trastuzumab: a review of its use in HER2‐positive advanced gastric cancer. Drugs 73, 1605–1615.2405741610.1007/s40265-013-0119-y

[9] Qiu MZ , Li Q , Wang ZQ , Liu TS , Liu Q , Wei XL , Jin Y , Wang DS , Ren C , Bai L *et al* (2014) HER2‐positive patients receiving trastuzumab treatment have a comparable prognosis with HER2‐negative advanced gastric cancer patients: a prospective cohort observation. Int J Cancer 134, 2468–2477.2415503010.1002/ijc.28559

The article "Trastuzumab induces PUMA‐dependent apoptosis and inhibits tumor growth in gastric cancer" was retracted in 2023. Reasons: duplicated images; signs of a paper mill.

[10] Luque‐Cabal M , Garcia‐Teijido P , Fernandez‐Perez Y , Sanchez‐Lorenzo L and Palacio‐Vazquez I (2016) Mechanisms Behind the Resistance to Trastuzumab in HER2‐Amplified Breast Cancer and Strategies to Overcome It. Clin Med Insights Oncol 10, 21–30.2704215310.4137/CMO.S34537PMC4811269

[11] Fleeman N , Bagust A , Beale S , Dwan K , Dickson R , Proudlove C and Dundar Y (2015) Pertuzumab in combination with trastuzumab and docetaxel for the treatment of HER2‐positive metastatic or locally recurrent unresectable breast cancer. Pharmacoeconomics 33, 13–23.2513817110.1007/s40273-014-0206-2

[12] Maly JJ and Macrae ER (2014) Pertuzumab in Combination with Trastuzumab and Chemotherapy in the Treatment of HER2‐Positive Metastatic Breast Cancer: Safety, Efficacy, and Progression Free Survival. Breast Cancer (Auckl) 8, 81–88.2485537210.4137/BCBCR.S9032PMC4022699

[13] Gao J and Swain SM (2016) Pertuzumab for the treatment of breast cancer: a safety review. Expert Opin Drug Saf 15, 853–863.2698234910.1517/14740338.2016.1167185

[14] Tong J , Wang P , Tan S , Chen D , Nikolovska‐Coleska Z , Zou F , Yu J and Zhang L (2017) Mcl‐1 Degradation Is Required for Targeted Therapeutics to Eradicate Colon Cancer Cells. Cancer Res 77, 2512–2521.2820251410.1158/0008-5472.CAN-16-3242PMC5626525

[15] Yang S , Zhu Z , Zhang X , Zhang N and Yao Z (2017) Idelalisib induces PUMA‐dependent apoptosis in colon cancer cells. Oncotarget 8, 6102–6113.2800814910.18632/oncotarget.14043PMC5351616

[16] Tong J , Tan S , Zou F , Yu J and Zhang L (2017) FBW7 mutations mediate resistance of colorectal cancer to targeted therapies by blocking Mcl‐1 degradation. Oncogene 36, 787–796.2739933510.1038/onc.2016.247PMC5226932

[17] Sun J , Knickelbein K , He K , Chen D , Dudgeon C , Shu Y , Yu J and Zhang L (2014) Aurora kinase inhibition induces PUMA via NF‐kappaB to kill colon cancer cells. Mol Cancer Ther 13, 1298–1308.2456354210.1158/1535-7163.MCT-13-0846PMC4013266

[18] Tong J , Tan S , Nikolovska‐Coleska Z , Yu J , Zou F and Zhang L (2017) FBW7‐dependent Mcl‐1 degradation mediates the anticancer effect of Hsp90 inhibitors. Mol Cancer Ther 16, 1979–1988.2861976010.1158/1535-7163.MCT-17-0032PMC5587378

[19] Gurzov EN , Germano CM , Cunha DA , Ortis F , Vanderwinden JM , Marchetti P , Zhang L and Eizirik DL (2010) p53 up‐regulated modulator of apoptosis (PUMA) activation contributes to pancreatic beta‐cell apoptosis induced by proinflammatory cytokines and endoplasmic reticulum stress. J Biol Chem 285, 19910–19920.2042130010.1074/jbc.M110.122374PMC2888402

[20] Peng R , Tong JS , Li H , Yue B , Zou F , Yu J and Zhang L (2013) Targeting Bax interaction sites reveals that only homo‐oligomerization sites are essential for its activation. Cell Death Differ 20, 744–754.2339212310.1038/cdd.2013.4PMC3619242

The article "Trastuzumab induces PUMA‐dependent apoptosis and inhibits tumor growth in gastric cancer" was retracted in 2023. Reasons: duplicated images; signs of a paper mill.

[21] Tong JS , Zhang QH , Huang X , Fu XQ , Qi ST , Wang YP , Hou Y , Sheng J and Sun QY (2011) Icaritin causes sustained ERK1/2 activation and induces apoptosis in human endometrial cancer cells. PLoS ONE 6, e16781.2140814310.1371/journal.pone.0016781PMC3050810

[22] Tong JS , Zhang QH , Wang ZB , Li S , Yang CR , Fu XQ , Hou Y , Wang ZY , Sheng J and Sun QY (2010) ER‐alpha36, a novel variant of ER‐alpha, mediates estrogen‐stimulated proliferation of endometrial carcinoma cells via the PKCdelta/ERK pathway. PLoS ONE 5, e15408.2107981110.1371/journal.pone.0015408PMC2973969

[23] Bean GR , Ganesan YT , Dong Y , Takeda S , Liu H , Chan PM , Huang Y , Chodosh LA , Zambetti GP , Hsieh JJ *et al* (2013) PUMA and BIM are required for oncogene inactivation‐induced apoptosis. Sci Signal 6: ra2010.1126/scisignal.2003483PMC375358523532334

[24] Ren D , Tu H‐C , Kim H , Wang GX , Bean GR , Takeuchi O , Jeffers JR , Zambetti GP , Hsieh JJ‐D and Cheng EH‐Y (2010) BID, BIM, and PUMA are essential for activation of the BAX‐and BAK‐dependent cell death program. Science 330, 1390–1393.2112725310.1126/science.1190217PMC3163443

[25] Chen D , Wei L , Yu J and Zhang L (2014) Regorafenib inhibits colorectal tumor growth through PUMA‐mediated apoptosis. Clin Cancer Res 20, 3472–3484.2476361110.1158/1078-0432.CCR-13-2944PMC4079733

[26] Holohan C , Van Schaeybroeck S , Longley DB and Johnston PG (2013) Cancer drug resistance: an evolving paradigm. Nat Rev Cancer 13, 714–726.2406086310.1038/nrc3599

[27] Housman G , Byler S , Heerboth S , Lapinska K , Longacre M . Longacre M , Snyder N and Sarkar S (2014) Drug resistance in cancer: an overview. Cancers (Basel) 6, 1769–1792.2519839110.3390/cancers6031769PMC4190567

[28] Kerbel RS (2001) Molecular and physiologic mechanisms of drug resistance in cancer: an overview. Cancer Metastasis Rev 20, 1–2.1183163610.1023/a:1013129128673

[29] Periti P and Mini E (1989) Drug resistance in cancer: an overview of the clinical aspects. J Chemother 1, 5–9.10.1080/1120009x.1989.117388562656931

[30] Carpenter RL , Han W , Paw I and Lo H‐W (2013) HER2 phosphorylates and destabilizes pro‐apoptotic PUMA, leading to antagonized apoptosis in cancer cells. PLoS One 8, e78836.2423605610.1371/journal.pone.0078836PMC3827261

[31] Zheng X , He K , Zhang L and Yu J (2013) Crizotinib induces PUMA‐dependent apoptosis in colon cancer cells. Mol Cancer Ther 12, 777–786.2342729410.1158/1535-7163.MCT-12-1146PMC3651803

[32] Dudgeon C , Peng R , Wang P , Sebastiani A , Yu J and Zhang L (2012) Inhibiting oncogenic signaling by sorafenib activates PUMA via GSK3beta and NF‐kappaB to suppress tumor cell growth. Oncogene 31, 4848–4858.2228675810.1038/onc.2011.644PMC3342476

The article "Trastuzumab induces PUMA‐dependent apoptosis and inhibits tumor growth in gastric cancer" was retracted in 2023. Reasons: duplicated images; signs of a paper mill.

[33] Sun J , Sun Q , Brown MF , Dudgeon C , Chandler J , Xu X , Shu Y , Zhang L and Yu J (2012) The multi‐targeted kinase inhibitor sunitinib induces apoptosis in colon cancer cells via PUMA. PLoS ONE 7, e43158.2291281610.1371/journal.pone.0043158PMC3422222

